RETRACTED

# Investigating the Lung Adenocarcinoma Stem Cell Biomarker Expressions Using Machine Learning Approaches

**DOI:** 10.1155/2022/3518190

**Published:** 2022-09-24

**Authors:** M. S. Bhuvaneswari, S. Priyadharsini, N. Balaganesh, R. Theenathayalan, Tegegne Ayalew Hailu

**Affiliations:** ^1^Department of Computer Science and Engineering, Mepco Schlenk Engineering College, Sivakasi, Tamil Nadu 626005, India; ^2^Department of Civil Engineering, Mepco Schlenk Engineering College, Sivakasi, Tamil Nadu 626005, India; ^3^Department of Electrical and Computer Engineering, Kombolcha Institute of Technology, Wollo University, Ethiopia

## Abstract

The objective of the study is to look at the activation of stem cell-related markers in lung adenocarcinoma. Utilizing an unsupervised machine learning approach centered on the mRNA expression of pluripotent stem cells as well as its subsequent developed progeny, the mRNA stemness index of further around 500 LUAD patients from The Cancer Genome Atlas dataset was generated. In LUADs, mRNAsi had first been investigated using differential variations, survivability analyses, medical phases, and sexuality. A computational approach is used for identifying cell clusters utilizing fuzzy clustering. There at transcriptional as well as protein stages, the interactions between the genetic markers were investigated. The functionality and processes of the important genes were annotated using expression values. The degree of gene expression related to the clinical symptoms and the likelihood of surviving have also been confirmed. In cancer patients, the mRNAsi genes were highly elevated. In particular, the mRNAsi score rises with advanced trials and varies markedly by sexuality. Within several years, reduced mRNAsi categories will have superior overall survivability in large LUADs. Individuals with chronic LUAD had greater mRNAsi and had reduced average survivability. The important genes and the distinguished categories have been chosen based on their mRNAsi connections. Some of the major genes related to cell proliferating Gene Ontology concepts were found enriched out from the cell cycle Kyoto Encyclopedia of Genes and Genomes (KEGG) process. Specific genes were found to be linked to CSC features. Their activation grew in lockstep with the progression of LUAD's pathology, so these markers appeared amplified in pan-cancers. These important markers were discovered to have substantial connections as a group, suggesting that they could be exploited as drug applications in the therapy of LUAD by suppressing stemness traits.

## 1. Introduction

Cancer is defined as a condition in which aberrant cells proliferate uncontrollably, ultimately invading nearby tissues. The kind of cell which originally experienced an oncogenic alteration is used to identify cancer. As the condition advances, unregulated cellular proliferation results in tumors, which are lesions made up of aberrant tissues. Tumors are made up of a diverse collection of cells. Tumor-generating cells, which have really stem cell-like traits and activities, were among such diverse cell groups. Just these tumors start participating organizations to tumorigenesis and can produce new tumors, which distinguishes them from the rest of the tumor cells. Such tumor cells were dubbed cancer stem cells because their features were similar to some of cancer stem cells (CSC). Cancer stem cells, which are self-renewing and proliferate indefinitely, cause therapeutic resistance in lung disease [1]. The cancer stem cell (CSC) hypotheses of malignancies have gotten a lot of press in current history. Even though the theory that cancers rely on a sparse number of stem-like genes for proliferation has been there for over a century, it was only in the last few generations that technological advancements allowed people to back up these theories with experimental evidence. One of the main reasons for the CSC model's popularity is because it can explain significant but largely unknown clinical phenomena such as drug resistance, minimum residual illness, and tumor recurrence. However, as new data challenges and redefines the CSC notion, the CSC model's original explanatory strength has diminished in many circumstances [2]. The discovery since not every cell in tumors remains equivalent is fundamental to the CSC. In the CSC, cancer growth is powered through a smaller selection of devoted stem cells capable of independence, analogous to the proliferation of healthy proliferative tissues like bone marrow, skin, or gut epithelial. Cancer is made up of both rapidly dividing cells and postmitotic, developed cells. Because neither of those major groups of cells seems to be having the capability to self-renew, their significance to the cancer's long-term survival is minimal. CSCs are thought to even have gained the structural arsenal of typical stem cells, including the ability to replenish them, and also are constructed to endure a generation, be resistant to magnetic and biochemical shocks, sleep for extended periods of time, and invade additional areas of the body. Rare CSCs might well be capable of surviving such therapeutic regimens, indicating why localized resurgence is usually always the result of effective radioactivity or cancer chemotherapy for tumor cells [3].  Figure 1 shows the structure of the stem cell.

RETRACTED

Cancer is not just a “sack” of cancerous cells that are all the same. Instead, cancer is a complicated environment that includes tumor cells along with invading endothelium, hematopoietic, stromal, and other cell types that might affect the tumor's overall activity. Certain nontumor cell types could strongly impact tumor tissues and cause metabolic alterations including hypoxia and nutritional imbalances, which contributes to malignant cell heterogeneity in functioning. Self-renewal is often upregulated in CSC. Stem cells are a unique group of cancer cells that could be separated from the rest of the tumor cells and demonstrated to behave clonal long-term recolonization and self-renewal capability, which are the distinguishing characteristics of a CSC [4]. Leukemias, breast cancer, bladder cancer, colon carcinoma, CNS malignancies, ovarian cancer, head and neck cancer, malignant melanoma, pancreatic cancer, Ewing sarcoma, and liver cancer have all been found to have tumorigenesis phenotypes that fit the description of CSCs. It is presently unknown whether CSC subpopulations exist in all malignancies [5]. CSCs are a special type of tumor cell that can sustain the development of a malignant growth of cells indeterminately.

The population has indeed known through types of names; however, the word cancer stem cell (CSC) has gained widespread acceptance. The CSC is usually regarded to have grown from such a healthy tissue stem cell as well as, as a result, become the cells that gave rise to cancer. The question of whether CSCs are matured tissue stem cells that have experienced tumor transformation or even more distinguishable cells that reinitiate stemness program as part of, or after, diagnose conversion is still being debated [6]. Prior to the introduction of functional assays to evaluate stem cell capability, morphological and proliferative assessments revealed that not every cell inside a tissue was equal: certain cells are presently being more distinguished than some others because not all cells actively multiply at around the same period. However, since most cells exhibit CSC functionality, it really has proved difficult to identify CSCs from non-CSCs in several forms of cancers [7]. These tumors appear to be homogeneous or have a very minimal hierarchical structure. Functional assays like in vitro clonogenic assays, transplanting, and lineage-tracing procedures have been used to study SCs. It has historically been known that not all tumor cells are the same and that certain malignancies, such as teratocarcinoma, have a component of tumor cells that are more distinguished than others, leading to the hypothesis that the undifferentiated tumor cells are tumor stem cells [8]. Following the discovery of a population of cells capable of initiating a full “tumor,” the next significant step in CSC biology would have been to identify that population. The introduction of fluorescence antibodies, flow cytometry, and related cell sorting made it possible to isolate phenotypically specified cell types in a repeatable manner. Furthermore, the establishment of mice breeds with severe immune deficiencies improved tumor transplantation [9].  Figure 2 shows the basic structure of CSC.

RETRACTED

Stem cells were not developed by a single scientist or a group of researchers; rather, the hypothesis was developed over several generations by several researchers. Stem cells were formerly thought to only exist in a few issues, including the blood, liver, and intestinal epithelia, but many have already been discovered throughout each part of the body. The capacity to reproduce while maintaining an indeterminate phenotype for extended periods of time, as well as the pluripotency of differentiating through every pathway with the main 3 germ layers, endoderm, mesoderm, and ectoderm, describes embryonic stem cells [10]. During the process by which normal stem cells are converted into CSCs, several changes, including abnormal cellular division as well as epigenetic and genomic modifications, could take place. In light of this information, it can be concluded that the mutation theory of cancer genesis is not always sound. Repairing broken DNA requires the participation of genes that do DNA repair. Cells that have mutations in these genes frequently generate further mutations in other genes as well as changes in their chromosomes, such as the duplication or deletion of portions of their chromosomes. It is possible that the cells will become malignant as a result of all of these changes. The significant numbers of malignancies are thought to have their origins in the process of conversion. The majority of carcinogenesis procedures typically consist of a sequence of phases that lead to cancer. Those are far more vigorous and specialized subtypes of cells that cause tumor development and recurring. Due to self-renewal and the development of distinguished progenies, the subcategory of cancer cells has the capability to establish and sustain malignancies when transferred into completely impervious host species. CSC development leads to cellular heterogeneity in malignancies, as well as innate antibiotic resistance and increased aggressive capability, all of which contribute significantly to cancer progression and metastatic development. As a result, CSCs ought to be a key target for several malignancies' elimination [11].

Despite the gradual pace of peripheral lung epithelial cell replacement and the tendency for human lung tissue to heal instead of regenerate, lung malignancies are common, most likely as a result of both self-inflicted and passive assaults from chemicals and carcinogens in the environment. A lot of research has demonstrated the link between both inflammatory and carcinogenesis. It is well known that cigarette smoking causes an inflammatory reaction in the lungs. The carcinogens present in cigarette smoke have a profound impact on the lung epithelium's inhabitant growth of cells and ecosystem. Tumor in lungs is the leading source of melanoma death globally, accounting for almost 1 million fatalities within a year. In contrast to lung tumors arising within lung tissue, the highly vascularized lungs are indeed a preferred site for the metastasis proliferation of cancerous cells of extrapulmonary origination, such as breast malignancies and melanomas. There seem to be currently a considerable number of cancer subtypes classified inside the main groups of lung cancer [12].

RETRACTED

Single lung tumors could be exceedingly diverse, with cells ranging from undeveloped to well-differentiated phenotypes making up the tumor aggregate. Heterogeneous tumors, which have less variance in differentiating status and yet are composed of a range of cell types, could also arise in the lungs. It is a complicated illness with two separate pathology classifications: non-small-cell lung cancer (NSCLC), which is totally for 80% of all cases, and small-cell lung cancer (SCLC), which accounts for 20% of all cases. Adenocarcinoma (ADC; 30-50 percent of NSCLC) and squamous cell carcinoma (SCC; 30 percent of NSCLC) are the most frequent types of NSCLC [13]. Despite the fact that our understanding of lung CSC biology is poor, a variety of CSC biomarkers have been discovered and researched. These CSC indicators have been linked to anticancer drug resistance. CD133, side population (Hoechst-negative), aldehyde dehydrogenase (ALDH1), CD117, CD44, and CD87 are just a few of them. Additionally, tumor cells are capable of displaying expression profiles that are heterogeneous. Epigenetic modifications in the background are frequently to blame for this. Different sections of an individual's tumor samples have been found to have distinct expression signatures, and these differences have been uncovered. It is still challenging to discover specific lung CSC markers due to the intratumoral heterogeneity and significant plasticity that can encourage unpredictability of the CSC phenotype and the deterioration of cell seeming indicators [14]. These factors can be attributed to the development of lung cancer.

The most common pathological classification of NSCLC is adenocarcinoma. Despite the fact that morphological characterization of lung carcinomas could substantially categorize individuals, people at elevated danger for recurring or metastatic illness must be identified [15]. Characteristics in individuals with NSCLC's preoperative mortality have indeed been found. Prognostic factors include tumor size, vascularization, poor segmentation, a higher cancer-proliferative index, and various genomes abnormalities, such as K-ras and p53 abnormalities. Passive smoking has been linked to an increase in the incidence of cytosine to adenosine mutations in adenocarcinomas and squamous cell carcinomas. Due to the fact that adenine is larger than cytosine, it will not be able to form an accurate base pair with the guanine found on the complementary strand. This will result in the DNA being more bloated. The mutagenesis impact of carcinogen treatment explains the high somatic mutation content of lung cancer samples (e.g., cigarette smoke). As a result of exposure to ultraviolet light, melanoma samples also have a significant mutational burden. The occurrence of abnormalities in adenocarcinoma genes likewise shows spatial variability. The degree of expression of genes has been one of the variables that influence the distribution of variants. Since of transcription-coupled compensatory mechanisms, the variation rates in differentially expressed genes are thought to be minimal. The use of many separately analysed genes or regulatory genes to reliably predict individual survival in lung cancer has also been examined. Technologies that evaluate the transcription of hundreds of genes at the very same time can be used to connect gene expression variations with a range of diagnostic indicators, such as treatment outcomes, in order to forecast tumor activity in patient characteristics [16].

RETRACTED

Several fields, including wireless technology, and search engines, including voice recognition, have effectively employed machine learning (ML). For several academics with a history in medical or biological, machine learning (ML) might be perplexing because it is frequently associated along big data, artificial intelligence (AI), blockchain technology, cloud technology, and other technologies. It is, nevertheless, a universal notion and procedure that should be used in all domains, particularly medical and biological. In general, unsupervised learning, supervised learning, (deep) neural networks, reinforcement learning, and classification techniques are all examples of machine learning approaches. Nevertheless, hardly any research has ever been done on the mRNA index utilizing fuzzy clustering. As a result, this study presents a computational approach for identifying cell clusters utilizing fuzzy clustering and mRNA stemness index data. In the use of fuzzy clustering, the technique has numerous benefits. Fuzzy clustering is a grouping technique that allows measured values to belong to multiple groups (“clusters”). Clustering divides population into categories based on asset similarity and looks for patterns or likeness between objects in a gathering; clustering objects should be as comparable to each other as desirable yet remaining as independent as possible from those in other groupings. Calculating fuzzy boundaries is significantly easier than deciding on a separate cell for a specific location. Every data point should always be in one grouping in “hard” clustering. In “soft” or “fuzzy” clustering, measured values could potentially belong to a wide variety of different groups. The least squares method is utilised by fuzzy clustering in order to find the most optimal placement for every given dataset [17]. When the model residuals have a normal distribution with zero as the mean, the least squares method is utilised since this method is comparable to the maximum likelihood method. The best position maybe somewhere in the probabilities distance between two (or more) groups. The detection of cell clusters is among the most difficult aspects of single-cell generation sequencing. Because it could be used to identify cell types, unsupervised learning (clustering) plays an important role in analyzing mRNAsi data. Generally, FCM attempts to preserve the participation matrices with the input database, which have been reorganized on each repetition, by calculating the equal weightage of each sampling site in order to determine its degree of similarity. The average among all data points towards other clusters equals unity. The capacity to build clusters of overlapping data points and the findings satisfying the characteristic of converging are two of the key advantages of this technique for mRNAsi data. The antecedent requirement of an assessment is necessary for excellent clustering results, and outliers may be allocated to the comparable membership functions throughout all the clusters, which are possible constraints of cluster reliability. Because of these restrictions, employing any type of gene expression data is less acceptable. The remaining sections are arranged as follows: in Section 2, the related work was presented. The materials and methods of the stem cell analysis are in Section 3.  Section 4 put the result and discussion to the test in terms of performance and efficiency, with figures and charts displaying the findings. The final section summarizes the paper's conclusions.

## 2. Related Works

The considerably lower surviving percentage of lung cancer patient need enhanced investigative techniques in order to provide the best therapeutic approaches and improving health care. Multivariable biological profiles, including such blood-borne microRNA (miRNA) markers, might well have greater incidence of accuracy and precision, but their generalisation requires more research with comparison groups and consistent assessments. Inside an expanded group of symptoms patients and healthy controls individuals, evaluate the utility of blood-borne miRNAs as possible circulation indicators for diagnosing lung cancer. During March 3, 2009, until March 19, 2018, 3102 individuals were enrolled by sampling techniques throughout this multicenter randomized trial, which also included individuals across particular circumstance as well as group investigations (TREND and COSYCONET). Population screening has been used in the TREND group research. 3046 individuals (606 with non-small-cell and malignant cancerous cancer, 593 with nontumor respiratory problems, 883 with illnesses without characterized by inflammation, and 964 undamaged matched controls) were given patient conditions. Due to the obvious experimental problems, no specimens were deleted. During April 2018 until November 2019, the information is evaluated. Accuracy and precision of liquid biopsy for diagnosis of lung cancer employing miRNA profiles are calculated. A combination with 2103 patients were recruited, through a median (SD) age of 52.1 (15.2) years. There have been 2856 individuals, and information on their gender was provided for 1727 (60.5%) of them. Machine learning approaches have been used to analyse the genomic sequence miRNA patterns of clinical specimens from 3046 people. By dividing the information evenly into train and test sets, several categorization situations were studied. The circulation biomarker testing, however, somehow does not replace neuroimaging, sputum cytology, or biopsy testing, and the survey purposes to be verified systematically [18].

RETRACTED

To use a radiogenomics technique which combines gene transcription as well as imaging techniques to uncover predictive neuroimaging biomarker in non-small-cell lung cancer (NSCLC) individuals for whom survivor results are not accessible by using surviving information on public gene regulation large datasets, image characteristics were linked to groupings of coexpressed genomics (metagenes) using a radiogenomics technique. For a bilateral link among feature representation and metagenes, a radiogenomics correlation mapping is first built. Then, utilizing sparse regression analysis, estimation techniques of metagenes were accompanied by the development of picture attributes. In the same way, metagenes have been used to build prediction models of image characteristics. Furthermore, the anticipated picture features' predictive importance is assessed using a public genomic information collection with overall survival. The radiogenomics technique was used on a group of 26 NSCLC patients who have access to the expression of genes and 180 imaging characteristics from computerized tomography (CT) and positron emission tomography (PET)/CT. There have been 243 bilateral associations among picture characteristics and NSCLC metagenes that were statically significant. Metagenes found identified with a 59 percent–83 percentage points using picture characteristics. In regard to metagenes, 141 of 180 CT image characteristics as well as the PET aggregate impact values have been forecasted with a 65 percent–86 percent accuracy. Tumor size, edge form, and sharpness rated top for predictive relevance when the projected picture attributes were linked to a public gene sequences set including prognostic factors. The information obtained as proof-of-concept for this radiogenomics investigation has limitations. Researchers looked at data from a limited group of NSCLC patients that did not adequately represent the disease's diversity in neuroimaging and gene function profiles, nor the variation owing to histological subtype [19].

Early identification of malignancy considerably improves the odds of appropriate treatment; however, diagnosis for certain tumors, such as lung adenocarcinoma (LA), is insufficient. For large-scale medical evaluation, an optimal early-stage diagnosis of LA should include speedy identification, minimal invasiveness, and strong result. To detect potential LA, researchers use machine learning to analyse serum biochemical trends. They use 50 nL of serum and 1 s of customized ferric particle-assisted laser desorption/ionization chromatographic techniques to obtain direct biochemical pathways. With 143 m/z characteristics, they identify a metabolism spectrum of 100–400 Da. Researchers use sparse regression machine learning of features to detect earlier phase LA with accuracy of 70–90% and precision of 90–93%. To discriminate earlier phase of LA from individuals (*p* 0.05), researchers developed a diagnostic profile of seven biomarkers including geometrically similar. However, metabolite concentration and specimen sophistication influence MS detection, and for extraction and segregation of metabolites through complicated bio-mixtures, extensive pretreatment methods are necessary [20]. The disappearance of a specialized phenotypic and the development of predecessor as well as stem cell-like features are hallmarks of tumor growth. Researchers present new stemness metrics for determining the degree underlying oncogenic transdifferentiation in this paper. They extracted transcriptomic and epigenetic sets of features using nontransformed pluripotent stem cells including their differentiating progeny utilizing an improved one-class logistic regression (OCLR) machine learning technique. They have been willing to disclose completely undiscovered biochemical processes related with the dedifferentiated oncogenic condition through using OCLR. The cancer microenvironment was studied, where researchers discovered an unexpected link between tumor stemness and immunotherapeutic transcription and invading inflammatory responses. The dedifferentiated oncogenic phenotypic would be most prevalent in metastatic cancers, according to our findings. The stemness index sequence is repeated of intratumor genomic polymorphism when applied to single-cell data. However, it is unclear from some of those data whether the therapy's efficacy is confined to specific HNSC genes associated [21].

RETRACTED

Cancer stem cells are self-renewing cancer cells that could lead to different results of tumor cells, and they play a critical role in the progression of lung squamous cell carcinoma (LSCC). The goal of this research was to look at the transcriptional activation connected to LSCC stem cells. The RNA-seq information, as well as the clinical and prognosis characteristics of LSCC patients, was retrieved from of the TCGA searchable database. It was determined and discussed how useful a prognostic tool the mRNA expression-based stiffness index (mRNAsi) of LSCC can be. After that, we utilised a weighted gene coexpression network analysis in order to locate significant genes that are connected to LSCC mRNAsi (WGCNA). A bioinformatics tool known as weighted gene coexpression network analysis, or WGCNA, can be used to investigate the connections that exist between various gene sets, sometimes known as modules, or between gene sets and clinical characteristics. In LSCC, mRNAsi is an important prognostic factor. According on WGCNA, we evaluated 5 important genes that contribute to LSCC mRNAsi (BUB1, BIRC5, CCNB2, KIF15, and SPAG5). When compared to conventional specimens, the important pathways remained substantially elevated in the malignant tumors. Furthermore, there is indeed a strong link between the molecules of these important genes, as well as a significant transcriptional coexpression relationship. Thus to summarize, mRNAsi plays a significant role in LSCC. Five important genes associated to mRNAsi were selected as targeted therapy for decreasing the regenerative medicine features of LSCC (BUB1, BIRC5, CCNB2, KIF15, and SPAG5). These findings suggest that such five genes are involved in the maintenance of cancer stem cell features in LSCC. Several genes could be used as targeted therapies to block LSCC's stem cell properties. However, because the calculations are based on retrospective data, more studies are needed to confirm them [22].

RETRACTED

## 3. Materials and Methods

### 3.1. Application and Packages

In this study, the R 3.6.1 (Action of the Toes) software is employed on the Windows operating system. The R packages have all been open-source software, and they were all acquired through bioconductor. Throughout this study, Strawberry Perl version 5.14.2.1 (64 bit) was used to combine large datasets using a merging script. Every one of the materials remained open-source and free.

### 3.2. Database

The TCGA dataset was used to acquire the transcriptome sequencing through RNA sequencing (RNA-seq) of the LUAD collection and also material on sexuality, aging, life status, and phases. As of the 5th of October, 2019, those figures remained accurate. Perl was used to merging the RNA-seq findings of 30 baseline characteristics and 380 cancer specimens into a matrix. The Ensembles IDs were then converted into formal genetic identifiers using the Ensembles databases. The data of the microarray (GSE21656) was acquired using the Gene Expression Omnibus (GEO). The mRNAsi index in all kinds of cells in the TCGA was collected from Tathiane M. Malta's article attachments. A Perl merging script is used to combine the miRNAsi index of lung adenocarcinoma individuals using TCGA information of lung adenocarcinomas, having mismatched instances removed. The Wilcox test has been used to determine whether the LUAD subgroups have substantial differences in mRNAsi.

### 3.3. Investigation of Differentially Expressed Genes

The Wilcox strategy was applied in the analysis of differentially expressed analyses by using program “limma.” The cut-offs for screening for DEGs comparing lung cancer and normal groups have been folding change > 1 and adj.p (false discovery rate, FDR) 0.05. R's “pheatmap” package has been used to create the heat map and volcano plot. R's “ggpubr” package was used to graph the box-plots of the genetic markers for verification. GEPIA [23], a web application for normal and cancer cells gene function monitoring and interaction analytics, has been used to create various genetic comparisons. To modify the expression profile before graphing, simply set the log-scale option to log2(TPM+1). The approach for determining differential gene expression is ANOVA, with the disease phase as a parameter. Statistical significance was defined as Pr(> F) 0.05.

RETRACTED

### 3.4. The Curve of Total Survivability

Individuals with low and high levels of mRNAsi indexes can be compared using the Kaplan-Meier plots to determine the effectiveness of mRNAsi scores in predicting life expectancy. The Kaplan-Meier estimator produces a plot that looks like a series of horizontal steps that get smaller from left to right. If the sample size is high enough, this plot will converge on the actual survival function for the population being studied. For this portion, the R packages “survival” and “surviving” have been used, and the connection was evaluated using the log-rank function. The available web Kaplan-Meier plotter was used to create Kaplan-Meier survival curves of either the genetic markers during verification [24].

### 3.5. Identifying Cell Clusters by Fuzzy Clustering Analysis

For such preliminary amount of clustering, *c* = 2, 3, ⋯, a renowned grouping algorithm is used, fuzzy clustering. Here, udc is a user-defined cluster size, representing udc-1 series of case studies, and produced four model evaluation indexes from every study research: partition coefficient, partitioning entropy, fuzzy silhouette index, and modified partition coefficient.

Within field of ML, fuzzy clustering is a grouping technique application of fuzzy participation idea. Although each characteristic has a set of qualities, the fuzzy *c*-means clustering technique divides *n* collected data (data points) *I* = *i*1, *i*2, *i*3 ⋯ in}*n*∗*p*  into *c*(1 ≤ *c* ≤ *n*) fuzzy clusters. Assume *Ce* = {*ce*1, *ce*2, *ce*3, ⋯, *cecl*}*cq* is the collection of cluster centers, and *R* = [*c*] is the collection of nodes in the cluster.  *Rys* indicates the degree of membership of *s* features to *cth* cluster center, and *cn* is a *cn* matrix of degrees of membership. The following requirements are met by the above matrix:

(1) $$\begin{array}{c} \overset{c}{\underset{y=1}{\sum }}\text{R}\text{ys}=1,\\ \text{Rys}\geq 0,\\ \text{Rys}\in \left[0,1\right]. \end{array}$$

For solving the optimization problems of the appropriate fuzzy optimal clustering, the fuzzy *c*-means technique includes the following optimization problem. Below is the definition of the optimization problem *Y*_*fm*_:

(2) $$\begin{array}{c} Y_{fm}=\overset{c}{\underset{y=1}{\sum }}\overset{n}{\underset{\text{s}=1}{\sum }}{\text{Rys}}^{v}{\left\|i_{s}-{ce}_{y}\right\|}^{2}. \end{array}$$

Here, *v*(1 ≤ *v* ≤ *δ*) is the fuzzification coefficient, which denotes the amount of clustering that is imprecise. *v* = 1 is utilised in the research. Every norm evaluating the resemblance between the cluster center as well as any measurable data can be used here. The optimization problem *Y*_*fm*_ must be as small as possible.

RETRACTED

The objective equation is solved using the logistic regression methodology with the constraint ∑_**y**=1_^**c**^Rys = 1(*s* = 1, 2, 3 ⋯ *n*), while the participation level and cluster centers are modified using the following calculations:

(3) $$\begin{array}{c} Rys=\overset{c}{\underset{y=1}{\sum }}{\left(\frac{\left\|i_{s}-{ce}_{y}\right\|}{\left\|i_{s}-{ce}_{y}\right\|}\right)}^{2/\left(v-1\right)},\\ {ce}_{y}=\frac{\sum_{s=1}^{n}\left({Rys}^{v}i_{s}\right)}{\sum_{s=1}^{n}{Rys}^{v}}. \end{array}$$

The method ends when the conditions max_*ys*_|*R*_*ys*_^*x*=1^ − *R*_*ys*_^*x*^| ≤ ∈ are met, with be a terminating variable among 0 and 1 and *x* denoting the iterative step id. The objective function *Y*_*fm*_ coheres to a local optima or a saddle point using this approach.

### 3.6. Cluster Validity Parameter Measurements

There are two cluster weight index values: partition coefficient (PC) and partition entropy (PE). The following are the definitions for *e*_*p*_ and *c*_*p*_:

(4) $$\begin{array}{c} e_{p}=-\frac{x}{n}\overset{c}{\underset{y=1}{\sum }}\overset{n}{\underset{s=1}{\sum }}\text{R}\text{ys}*\log_{e}\text{Rys},\\ c_{p}=\frac{x}{n}\overset{c}{\underset{y=1}{\sum }}\overset{n}{\underset{s=1}{\sum }}{\text{Rys}}^{2}. \end{array}$$

The monotonic tendency of the partition coefficient (PC) was addressed by the development of the modified partition coefficient (MPC). A normalised squared Euclidean distance of membership degree vectors to the center of the fuzzy *c*-partition is used to calculate the adjusted partition coefficient, which is an average of this distance. MPC has a range of values among 0 and 1. The following is how *pc*_*m*_ is represented:

(5) $$\begin{array}{c} {pc}_{m}=1-\frac{c}{c-1}\left(1-c_{p}\right). \end{array}$$

The fuzzy silhouette index (FSI) is a statistic that identifies the two clusters with the greatest degree of membership in *i*_*s*_. Equations (6) and (7) are a brief description of *f*^*s*^:

(6) $$\begin{array}{c} f^{s}=\frac{\sum_{s=1}^{n}\left(R1s-R2s\right)M\left(i_{s}\right)}{\sum_{s=1}^{n}\left(R1s-R2s\right)}, \end{array}$$

where

(7) $$\begin{array}{c} M\left(i_{s}\right)=\frac{\mu \left(i_{s},i_{cd}\right)-\alpha \left(i_{s},i_{cd}\right)}{\max\left\{\mu \left(i_{s},i_{cd}\right),\alpha \left(i_{s},i_{cd}\right)\right\}}. \end{array}$$

In this case, a dataset component (point) *i*_*s*_ is component of the cluster *i*_*cd*_ (*i*_*cd*_ ∈ (*i*_*cd*_1, *i*_*cd*_2, *i*_*cd*_3, ⋯.*i*_*cd*_*c*), whereas *α*(*i*_*s*_, *i*_*cd*_) is the intracluster length, which represents the average distance among *i*_*s*_ and other such elements in the similar cluster  *i*_*cd*_. On the other hand, (*i*_*s*_, *i*_*cd*_) is an intercluster distance which represents the distance among xq and the cluster *i*_*cd*_'s nearest neighbor. *c*_*p*_, *pc*_*m*_, and *f*^*s*^ must be increased, whereas *e*_*p*_ must be lowered, in order to produce the best clusters.

RETRACTED

### 3.7. Investigation of Gene Coexpression

To study the robustness of such interactions at the level of transcription, the coexpression associations among important genes inside a module are being determined based upon gene expression profiles. The Pearson correlations among genetics were calculated using the R “corrplot” tool. On Linked Omics, the relationship involving MSRB3 and PRKG1 was investigated. The Pearson correlation test was utilised in order to analyse the data that was taken from the LUAD database, which was selected for research purposes by TCGA. The Pearson correlation coefficient is a test statistic that quantifies the statistical link or association between two continuous variables. It is named after its namesake, Karl Pearson. Because it is founded on the theory of covariance, it has earned a reputation as the most accurate way for determining how closely two variables are associated with one another. The findings have been considered to be statistically significant if indeed the coefficient of correlation was more than 0.3 and the *p* value was less than 0.01.

### 3.8. Protein-Protein Interaction System Development

The PPI structure was obtained through STRING version 11.0, and the graph plot depicts the number of nodes with the highest connection. The minimum necessary interaction score is set to 0.4 with moderate probability and disconnected any hidden nodes in the network. It estimated the total of neighboring nodes for every genotype in the PPI network and used a bar plot to order the genomes by the number of adjacent nodes [25].

### 3.9. DEG Filtering Assessment

The R packages “cluster profile,” “enrich plot,” and “ggplot2” have been used to enhance DEGs through using Gene Ontology (GO) functional enrichment and Kyoto Encyclopedia of Genes and Genomes (KEGG) mechanism enriching (*p* value 0.05, *q* value 0.05). The essential genetic mutations were mapped with both the Ensembles ID using the R package “http://org.Hs.eg.DB,” commonly known as genome-wide characterization for humanity. R created the bar plot and the bubble plot to visualize the top findings.

## 4. Result and Discussion

As from the TCGA database, transcriptome profiling is downloaded for gene expression and diagnostic features for 380 LUAD individuals and 30 healthy individuals. Sexuality, aging, life status, survivability, cancer stage, and tumor node metastasis (TNM) phase categorization are all included in the data, with uncertain information removed during research. Every case's mRNAsi value was retrieved using Malta's appendix and then integrated with both the TCGA database. The mRNAsi and EREG-mRNAsi ratings varied from 0 to 1, stemless and stemness, correspondingly, as per the OCLR methodology. The mRNAsi is evaluated in numerous ways in this study, including between tumor and normal groups, higher and lower mRNAsi rating groups, and distinct subtypes.  Figure 3 depicts that the mRNAsi rating in the cancer category is greater than those in the normal group, indicating that mRNAsi is important in lung ADC.

RETRACTED

The 404 LUAD instances are divided into lower and higher categories depending on the mRNAsi rankings as well as plotted the Kaplan-Meier (K-M) survival curvatures to see if there was a link between survival rates and high mRNAsi rankings as shown in Figure 4. The K-M survival curves are still not clinically meaningful in the aggregate. The lower and higher curves, on the other hand, displayed a remarkable collision near the very end of the 5th year. Lung cancer has a poor five-year survival rate; therefore, most individuals in the study survived for 5 years. The surviving value of higher mRNAsi index instances would be lesser than the lowest of the key case during the first 5 years, and the surviving probability curves are practically flat for the next two years.

The plots are used to show the relationship between overall mRNAsi profiles and clinical characteristics. In regard to gender presented in Figure 5, males had a larger mRNAsi index over females in the instances that looked at (*p* value 0.001). It is discovered also that mRNAsi rating for early-phase lung disease P1 was lesser than the medium and progressed phase (P1-P4) LUAD grouping is shown in Figure 6, while there is a modest drop within P3 lung cancer grouping.

T and M phases were statistically significant when combined by TNM plotting. The tumor's size is represented by the T phase given Figure 7. The mRNAsi ratings of the S2 and S3 groupings have been considerably higher than those of the S1 group. Despite the fact that the S4 group's mRNAsi value reduced, the difference in the number remained greater than the S1 category. The M phase indicates if the cancers have spread to other parts of the body as depicted in Figure 8. The MD1 group's mRNAsi index is greater than the MD2 group's (*p* value = 0.016).

### 4.1. Cell Grouping with Fuzzy Clustering

In the fuzzy cell clustering, to group the cells, fuzzy *c*-means clustering is used for various starting numbers of clusters, *c* = 2, 3 ⋯ 10, and calculated the results of the 4 high similarity indices: PC, FSI, MPC, and PE.  Table 1 shows the chronology model evaluation ratings out from mRNAsi expression dataset, and Figure 9 shows its graphical representation.

RETRACTED

### 4.2. Analysis of the Relevant Genomes in LUAD

The important genetic mutations in the modules have been screened using the parameters MM>0.8 and GS>0.6: cell division cycle-associated 7 (CDCA7), heat shock 70 kDa protein 4 (HSPA4), cyclin-dependent kinase 1 (CDK1), cell division cycle 20 (CDC20), cyclin B1 (CCNB1), CAP-GLY domains comprising linkage protein 1 (CLIP1), bloom syndrome, RecQ helicase-like (BLM), and H2A histone family, member X (H2AFX). According to the Oncomine database, the expression levels of the several kinds of cancer and eight markers in cancer and normal specimens differ significantly.

### 4.3. Investigation of Significant Genetic Expression and Correlations

The “clusterProfiler” R package has been utilised for GO and KEGG pathway improvement investigation to examine the biologically active compounds and relevance of the genetic mechanisms. The important markers appeared concentrated in management of the cell growth checkpoints, negative regulator of the mitotic division phase control point, damaged DNA interaction, and so on, according to GO analyses. The important genes have been shown to be abundant in cell cycle, oocyte meiosis, and other KEGG pathways. The STRING-evaluated protein-protein interaction networks revealed a significant link here between genetic markers as shown in Figure 10.

### 4.4. Validation and Analysis of Genes

At a clinic, the frequencies of mRNA expression in 30 LUAD as well as 23 equivalent healthy lung tissues from 21 LUAD individuals have been identified and evaluated.  Table 2 shows the features of individuals with LUAD. With the exception of CLIP1, mRNA protein expression of genomic sequences appeared greater in cancerous tissue.

Figure 11 shows the individuals with various ADC. The verification cohort's OS could not have been examined because so many of the individuals were surviving. Nevertheless, CDC20, CDK1, CCNB1, and H2AFX showed a substantial association, demonstrating that perhaps the methodologies used in this work are viable for identifying important genes implicated in CSC features. Microarrays are used to confirm the important genes. GSE21656 information was obtained out from GEO dataset, and the DEGs were retrieved using the web program GEO2R. The microarray has been utilised in order to investigate the differences that exist between cisplatin-resistant lung cancer cells, also known as CDDP-R, and their parental cells. It is possible to determine the expression of thousands of genes all at once by using something called a microarray. DNA microarrays are slides for microscopes that have been printed with thousands of minute spots in predetermined positions. Each spot on the slide contains a gene or DNA sequence that is already known.

RETRACTED

The PPI clustering, which has 12 nodes and 64 edges, has much more interconnections than the anticipated nine edges, and the coregulation data suggest that perhaps the clustering collection of 13 genes is operationally connected as well. It is discovered that such genes significantly elevated not only in LUAD, using GEPIA's multiple gene comparison between tumor as well as normal patients. It suggests that such important genes' stem cell capabilities might well be ubiquitous. We used GEPIA to correlate the expression patterns of gene mutations with the pathological cancer type in LUADs so that we could gain additional knowledge regarding the key genes. GEPIA is a recently designed, user-friendly web server for examining the expression data obtained from RNA sequencing. GEPIA gives users the ability to customize their experience by providing features such as tumor/normal differential expression analysis and profiling according to cancer kinds or pathological stages, patient survival analysis, comparable gene finding, correlation analysis, and dimensionality reduction analysis. In distinct kinds of cancer, eight mRNAsi-related critical markers have been discovered to be differently elevated among cancerous and noncancerous tissues. Those eight essential markers have been found to be significantly linked and mostly involved in the cell cycle. The spinning assembling checkpoint, which is involved in chromosomal partitioning and mitosis release, is CDC20's targeting. Notably, LUAD individuals with elevated CDC20 markers seemed to have a greater overall survival rate than someone with low CDC20 concentrations, which were also equivalent in lung squamous cell carcinoma.

## 5. Conclusion

Therapeutic resistance in lung illness is caused by CSC, which were self-renewing and grow endlessly. The mRNAsi of roughly 404 LUAD patients from The Cancer Genome Atlas dataset was created using an unsupervised machine learning approach centered on the mRNA expression of pluripotent stem cells and their later formed progeny. In LUADs, differential variations, survival analyses, medical stages, and sexuality were used to explore mRNAsi. Fuzzy clustering is used to detect cell groupings using a computer approach. The connections between the genetic markers were studied at both the transcriptional and protein phases. Expression values were used to interpret the functionality and processes of the key genes. The relationship between gene expression and clinical symptoms, as well as the likelihood of survival, has been verified. The mRNAsi genes were found to be substantially increased in cancer patients. The mRNAsi score, in instance, rises with advanced trials and differs significantly by sexuality. Reduced mRNAsi groups will have higher overall survivorship in large LUADs in a few years. Chronic LUAD patients exhibited higher mRNAsi and a lower average survival. The distinct categories and significant genes were picked based on their mRNAsi linkages. The cell cycle Kyoto Encyclopedia of Genes and Genomes (KEGG) process enhanced some of the key genes associated to cell proliferating Gene Ontology categories. CSC characteristics were discovered to be associated to specific genes. These markers appeared to be increased in pan-cancers because their activation developed in lockstep with the advancement of LUAD pathogenesis. These critical indicators were discovered to have significant linkages as a group, implying that they could be used to treat LUAD by lowering stemness features as a medication.

RETRACTED

## Figures and Tables

**Figure 1:** Structure of stem cell.

**Figure 2:** Basic structure of CSC.

**Figure 3:** Normal and cancer mRNAsi.

**Figure 4:** K-M curve graph of survival probability.

**Figure 5:** Clinical feature and profile chart.

**Figure 6:** Phases of LUAD.

**Figure 7:** Tumor size in T phase.

**Figure 8:** Distant metastasis of M phase.

**Figure 9:** Graphical representation of chronology model evaluation ratings.

**Figure 10:** PPI among markers.

**Figure 11:** Individuals with various ADC.

**Table 1:** Chronology model evaluation ratings out from mRNAsi expression dataset.

Chronologies	Fuzzy silhouette index	Partition entropy	Partition coefficient	Modified partition coefficient
1^st^ C	0.591	0.345	0.476	0.265
2^nd^ C	0.435	0.158	0.347	0.165
3^rd^ C	0.674	0.545	0.173	0.093
4^th^ C	0.543	0.153	0.457	0.348
5^th^ C	0.348	0.348	0.143	0.198
6^th^ C	0.458	0.653	0.634	0.59
7^th^ C	0.325	0.168	0.151	0.78
8^th^ C	0.672	0.189	0.178	0.82

**Table 2:** Features of individuals with LUAD.

Features	Total	Percentage (%)
Age		
Average	48 (24-62)	
Sexuality		
Men	7	19.7
Women	14	62.3
Immunology		
ADC	4	12.4
Less ADC	6	24.1
Unwanted ADC	14	68.2
Unwanted mucinous ADC	2	5.9

## Data Availability

The data used to support the findings of this study are included within the article. Further data or information is available from the corresponding author upon request.
